# Big Data Technology in the Macrodecision-Making Model of Regional Industrial Economic Information Applied Research

**DOI:** 10.1155/2022/7400797

**Published:** 2022-07-18

**Authors:** Kaiyan Lin

**Affiliations:** Shengda Economics, Trade and Management College of Zhengzhou, Zhengzhou 451191, China

## Abstract

In the era of Internet +, modern industry has developed rapidly, the network economy has promoted the great development of the industrial economy, and the traditional industrial economic statistics method has not been suitable for the development needs of modern enterprises. In today's society, it can be described as the era of big data, the use of big data technology for industrial economic statistics is needed for the development of industrial modernization, and it is also a new requirement for industrial economic statistics put forward by social development. With the wide application of Internet of Things, cloud computing, mobile Internet, remote sensing, and geographic information technology in the economic field, precise economic policies have gradually developed and matured. Especially for different industries in the regional economy, according to the big data in the region, the big data mining technology and analysis technology can be used to obtain the development situation and future trend of the industrial economy in a timely and effective manner. Applying big data technology to macrodecision of regional economic information is an effective way to make macrodecision of current economy. Based on this background, this paper proposes a macroeconomic decision-making method for regional industries based on big data technology. Using data mining technology, time series data analysis methods combined with artificial intelligence analysis, the development trend of regional industries is obtained, and then the development trend of the industry is obtained. Development makes macroeconomic decisions. Taking agriculture as an example, the most popular analysis of the price trend of a certain agricultural product provides an effective reference for the development strategy of this agricultural product. The results show that the method proposed in this paper can effectively apply big data technology to the macrodecision-making of regional industrial economy. And it has better promotion significance.

## 1. Introduction

With the development of Internet information technology and the continuous updating of digital information, the data in the Internet age are even more massive. The amount of data generated by all walks of life is growing exponentially, and data types are also various, for the transmission, storage, and analysis of data to put forward higher challenges. With the rapid development of big data technology and the use of sensors, video surveillance, distributed databases, and other tools and technologies, you can understand the production and operation of enterprises in real time in multiple ways. Accurate statistics of economic operation of enterprises can greatly improve work efficiency. The development of big data has challenged the epistemology established in science, social science, and humanities and has formed a paradigm shift in a multidisciplinary range [1]. The big data revolution has brought new challenges and opportunities to the traditional scientific epistemology; this change in thinking allows people to cleverly use data to understand and explore the world, inspire new products and services, and change our way of life, worldview, and thinking patterns [2]. Second, big data has brought about business changes [3]. Today, we can use data to create new economic benefits. Data have become an important business investment.

The extensive use of big data technology in the economic field ensures the timeliness of data information and provides more comprehensive and effective data for industrial economic information analysis [4]. Enterprises are in the process of development of a large number of data every day, the traditional data statistical analysis methods have not been able to keep up with the rhythm of the development of the times, and in the face of a vast sea of data, only the use of advanced big data technology for data statistical analysis work can improve work efficiency, while ensuring the accuracy of statistical analysis and enhancing the quality of analysis work. Efficient public services using big data to promote the transformation of government functions and improve the functions of government governance, while building a service-oriented government, is the issue that the government has always paid attention to and attached great importance to. With the continuous improvement of the application level, the national macrocontrol policy can be better implemented, and the economic control and decision-making methods can be effectively improved [5]. The steady growth of the industrial economy is of great significance to the stable operation of the macroeconomy and through a reasonable combination of policies, it can not only promote the steady growth of the current industry, but also cultivate and expand new kinetic energy, promote the optimization and upgrading of the industrial structure, and lay a solid foundation for the longer-term sustained and healthy development of the industry.

Based on this background, this paper studies the role of big data technology in macrodecision of regional industrial economic information, uses data mining technology to analyze industrial economic information, extracts the characteristics of industrial development, and provides guidance for macrodecision of regional economy.

## 2. State of the Art

Big data technology refers to the application technology of big data, covering all kinds of big data platforms, big data index systems, and other big data application technologies. Big data refers to collections of data that cannot be captured, managed, and processed with conventional software tools over a certain time frame. It is a massive, high-growth-rate, and diversified information asset that requires a new processing model to have stronger decision-making power, insight, and process optimization capabilities. Big data was first used to describe a large data set, which needs to be processed and analyzed in batches, and at the same time, the network-related indexes will be continuously updated [6]. It is very difficult to process and analyze these massive data by using existing database management tools [7].  Figure 1 shows the current framework for applying big data technology to the actual industry.

The current industry-recognized big data has the characteristics of “4V” (as shown in Figure 2) [8]. Big data 4V characteristics have a large amount of data: big data usually refers to the amount of data more than 100 tb. Wide variety of data means the important characteristics of big data are diverse and complex. Fast data processing speed means data are from generation to use, the time window is very small and can be used to generate decisions, and the time is very short. Low data value density means mining the value of big data is similar to panning for gold in the sand, mining sparse and valuable information from big data. Due to the large volume and diverse structure of big data, the value density created by it is significantly lower. It is only by summarizing massive data and using relevant processing technology, in order to effectively analyze and mine the value of data.

The industrial economic information model is mainly composed of seven subsystems, as shown in Figure 3 [9]. They are data information acquisition subsystem, knowledge base subsystem, information analysis subsystem, information contact and sharing subsystem, data processing subsystem, auxiliary decision-making subsystem, and information feedback subsystem. Various subsystems are interrelated and affect each other, and they work together to promote the normal operation of the entire model system. Therefore, the model has extremely high scalability, reliability, and fault tolerance [10].

Collect relevant information and combine the information outside the database to perform data integration processing to obtain new data information [11]. This can happen by analyzing the economic information of the industry, collecting the economic information of the industry in different periods, analyzing the past and current situation of the industry, and then predicting the future development of the industry. Scientific industrial economic information must be predictable to a certain extent, which can help enterprises to understand the development trend of the future market and then make economic decisions with more foresight and development significance [12].

Industrial macrodecision refers to the guidance and planning of major issues such as development goals, strategic measures, and implementation steps for each industry in the national economy at each stage of its life cycle. In the Internet era, the industry's analysis of economic data and information does not only stay in the traditional way, but analyzes financial and other transaction data and makes relevant trend forecasts, completes economic information analysis, and makes macrodecisions to ensure that they can obtain maximum benefits [13]. All departments of the industry can obtain the economic information they need from the database and make full use of it to conduct a comprehensive and systematic analysis to ensure that the information is effectively developed. At the same time, for the industry as a whole, the most important thing is to integrate the atmosphere of various departments, promote the coordinated progress of various departments, and ensure that economic information can be collected. In the era of big data, the analysis of industrial economic information has been comprehensively improved, and the accuracy and speed of macrodecision-making have been improved.

## 3. Methodology

The collected data are processed by the preprocessing technology, the data are stored through the big data storage and management technology and then also include the computing mode and system of big data, analysis, and mining technology, and finally the results obtained after a series of big data processing and analysis are presented using big data visualization technology [14]. It should be noted that big data security technology runs through the entire big data processing process. Taking the agricultural industry as an example, its process is shown in Figure 4.

### 3.1. Data Mining Technology

Data mining originated from and is oriented to applications. The most typical example is the discovery of the association between beer and diapers in a large supermarket chain [15], the feasibility of lending a user and the amount of loans. In short, data mining can be applied to all walks of life, and the knowledge can be used for information management, data maintenance, decision support, process control, etc. [16].

Data mining is the process of excavating information from massive data and guiding practice. It is a complete process that generally includes three stages: data preparation, data mining processing, and result interpretation and evaluation. This process is often repeated and approaches the essence of things until a solution to the target problem is found [17]. The complete process of data mining is shown in Figure 5.

#### 3.1.1. Data Preparation

Data preparation is an important link in the data mining process, and the entire preparation work consumes about 50%–90% of the time and energy of the entire data mining project. If the data preparation work is done well and the input data are of high quality, then the data mining modeling will be more convenient and fast, the mined patterns will be more effective and applicable, and the obtained results will have more practical guiding value. The entire data preparation stage includes data selection, data cleaning, and data transformation [18].

#### 3.1.2. Data Mining Processing

The data mining stage is the link that most analysts and researchers care about most. Data mining algorithms include classification analysis, cluster analysis, association analysis, and sequence analysis. The choice of algorithm directly affects the quality of pattern recognition [19]. Considering that data mining often serves ordinary users or scientific researchers, the selection of algorithms should also be closely combined with user needs.

#### 3.1.3. Interpretation and Evaluation of Results

Interpreting and evaluating results is an integral part of the entire data mining process. It can be seen that the entire data mining process is an iterative process until a solution to the target problem is found to meet customer needs [20].

### 3.2. Time Series Analysis

A time series, also known as a dynamic sequence, refers to a sequence formed by chronologically forming the statistical observations of the same indicator. As one of the quantitative forecasting methods, it includes general statistical analysis (such as autocorrelation analysis and spectral analysis); the establishment and inference of statistical models; and optimal forecasting, control, and filtering of time series.

Exponential smoothing refers to eliminating irregular fluctuations in historical statistical series in a certain way and finding out the development trend. If the fluctuation of the time series has stability or regularity, then the time series can be reasonably delayed. The simple moving average method is to use the past observations to calculate the predicted value of the next period, in which the number of past data points and data weights are unchanged, and each calculation iteration needs to remove the farthest observation value and add the nearest observation value at the same time. The formula for calculating the predicted value *y* is as follows:

(1) $$\begin{array}{c} y_{t+1}=\frac{x_{t}}{N}+\frac{x_{t-1}}{N}+\cdots +\frac{x_{t-N+1}}{N}\\ =\frac{1}{N}\sum_{t-N+1}^{t}x_{t},\\ y_{t+1}=\frac{x_{t}}{N}-\frac{x_{t-N}}{N}+y_{t}. \end{array}$$

The moving average has two main limitations: first, it needs to occupy a lot of memory space, because it needs to store a large number of past observations during prediction. The inner observations are given the same weight, and the weights of observations earlier than *N* periods drop sharply to zero. It can be seen that the exponential smoothing method is an improved method of the moving average method. If the data are stationary, replace *X*_t-N_ with the predicted value *y* of the previous period, as shown in

(2) $$\begin{array}{c} y_{t+1}=\frac{x_{t}}{N}-\frac{y_{t}}{N}+y_{t}\\ =\frac{1}{N}x_{t}+\left(1-\frac{1}{N}\right)y_{t}. \end{array}$$

The formula of the first exponential smoothing model is thus obtained as shown in

(3) $$\begin{array}{c} y_{t+1}=\alpha x_{t}+\left(1-\alpha \right)y_{t}. \end{array}$$

The second exponential smoothing method is to exponentially smooth the sequence data after one exponential smoothing. The first-order exponential smoothing model cannot well fit the sequences with obvious rising or falling trends. The second-order exponential smoothing is a method designed to make up for this defect. It has two parameters a and *T*, which is very suitable for analyzing the trend of sequentiality. The prediction model of the quadratic exponential smoothing method is as follows:

(4) $$\begin{array}{c} y_{t+\tau }=a_{t}+b_{t}\tau ,\\ a_{t}=2S_{t}^{1}-S_{t}^{2},\\ b_{t}=\frac{a}{1-a}\left(S_{t}^{1}-S_{t}^{2}\right),\\ S_{t+1}^{2}=\alpha S_{t+1}^{1}+\left(1-\alpha \right)S_{t}^{2}. \end{array}$$

It has been proved that the prediction accuracy of the second exponential smoothing method is higher than that of the first exponential smoothing method except for the sequence turning point. However, the quadratic exponential smoothing method is not suitable for dealing with periodic sequence data, and the quadratic exponential smoothing method has the problem of lag error. At this time, the triple exponential smoothing method is used, which is to exponentially smooth the sequence data after the second exponential smoothing.

### 3.3. Intelligent Analysis Method

In recent years, with the wide application of information technology and intelligent technology in various fields, intelligent data analysis refers to the use of statistics, pattern recognition, machine learning, data abstraction, and other data analysis tools to discover knowledge from data analysis methods. The purpose of intelligent data analysis is to directly or indirectly improve work efficiency, act as an intelligent assistant in practical use, enable staff to have the right information at the right time, and help them make the right decisions in a limited time. The artificial neural network is applied in the field of forecasting, and it mainly exerts its nonlinear mapping ability. The artificial neural network imitates the structure and functional characteristics of brain cells, establishes a mathematical model of nonlinear mapping, and inputs a large amount of historical data to learn the pattern pair.

The most basic unit of artificial neural network is artificial neuron, which forms different neural network structures through certain topological structures and algorithms. The goal of an artificial neuron is to determine the connection weights (weights) in it by training it on the input signal given the corresponding output signal. It is usually a nonlinear device with multiple inputs corresponding to a single output, and its structural model is shown in Figure 6.

The input vector of artificial neuron *j* is

(5) $$\begin{array}{c} X_{j}={\left(x_{1},x_{2},\ldots ,x_{n}\right)}^{T}. \end{array}$$

For each input *x*_*i*_(*i* = 1,2, ..., *n*), *n* represents the number of input artificial neurons. The input weight vector of each neuron can be expressed as

(6) $$\begin{array}{c} W_{j}={\left(w_{1j},w_{2j},\ldots ,w_{nj}\right)}^{T}. \end{array}$$

The actual output of the artificial neuron is the difference between the weighted vector sum and the threshold, and its formula can be expressed as

(7) $$\begin{array}{c} s_{j}=\sum_{i=0}^{n}x_{i}w_{ij}\\ =\sum_{i=1}^{n}x_{i}w_{ij}-\theta_{j}. \end{array}$$

## 4. Result Analysis and Discussion

Using the concepts, technologies, and methods of big data to process these agricultural data with extensive sources, complex structures, diverse types, and potential value, valuable information can be obtained to guide agricultural production, operation, circulation, and consumption of agricultural products. In order to measure the role of big data technology in the macrodecision-making model of regional industrial economic information, we select agriculture, a typical regional industry, for analysis.

### 4.1. Agricultural Big Data

Agricultural big data is a collection of data with a wide range of sources, diverse types, complex structures, and potential value, and it is difficult to apply the usual methods to process and analyze it after integrating the characteristics of agriculture, such as regionality, seasonality, diversity, and periodicity. There are five applications of agricultural big data: Reliable Decision Support System for Precision Agriculture, National Rural Comprehensive Information Service System, Agricultural Data Monitoring and Early Warning System (Price Forecast of Agricultural Products), Sky-Earth-Network Integrated Agricultural Conditions Monitoring System, and Agricultural Production Environment Monitoring and Control System. Agricultural big data production is an important stage in the development of agricultural modernization. The Reliable Decision Support System for Precision Agriculture can more effectively provide scientific planting guidance for agricultural practitioners. A large amount of raw data accumulated in the process of precision agriculture provides data guarantee for the analysis and processing of agricultural big data. At the same time, agricultural big data analysis provides technical support for agricultural product price prediction and can provide more accurate agricultural product price information services, thereby guiding agricultural practitioners to be reasonable. Planting agricultural products to achieve a win-win situation between producers and consumers thus forms a virtuous cycle and a closed-loop agricultural production chain from precision agriculture to agricultural big data to agricultural product price forecasting, as shown in Figure 7.

### 4.2. Basis for Macroeconomic Decision-Making of Industrial Economy

Within the framework of economic theory, market price fluctuations are reasonable adjustments to resource use and product production. Small market price fluctuations are a normal response to production adapting to demand. It is affected by many factors in supply and demand as well as the external environment. Price fluctuation is the objective law and self-adjustment of the market economy. Although price volatility is a normal economic phenomenon, if prices fluctuate too frequently or too much, it can have an impact on the income of producers and the lives of consumers. The price of agricultural products also has the above-mentioned fluctuation law, so for typical agricultural areas, macrodecision based on industrial economic information has important practical significance.

When the price of agricultural products is high, the farmers are more motivated to produce, and they will be planted in large quantities, which will increase the output of agricultural products, and the prices will drop accordingly. It affects the supply of agricultural products, which in turn affects the market price. Taking garlic as an example, as shown in Figure 8, it is generally planted in September and October and produced in May and June. In the cycle from garlic planting to output, farmers choose whether to plant and how much to plant in September and October. Regarding a decision point, May and June of the second year are the output points. In this process, the price of garlic at the output point has a very important influence on the decision-making of agricultural products at the decision point. Therefore, for the second year, May and June, the forecast of the garlic price at the point of production in the month is crucial.

It can be seen from this that knowing the price trend of agricultural products, through macroeconomic control, farmers can choose to increase or decrease the planting area reasonably and let farmers walk in front of market information, which can solve the problem of abundant supply of agricultural products and falling market prices. Regarding pressure, the price formation mechanism of agricultural products is the premise for analyzing the price fluctuations of agricultural products. From the equilibrium price and the cobweb theory, it can be seen that the market supply and demand force is the basis for the formation of a product price, and when the supply and demand force of the agricultural product market changes, it will lead to corresponding changes in the market price of agricultural products. Therefore, the price fluctuation of agricultural products is a normal phenomenon. Producers of agricultural products are easy to decide the current production decision based on the previous price information, thus generating the current market supply, while consumers usually determine the current market demand for agricultural products according to the current market price, which causes the price of agricultural products to be affected by the cycle of “supply and demand—price—supply and demand” which often shows the characteristics of cyclical fluctuations. In order to more accurately predict the price of agricultural products before and after the output point, many factors need to be considered. The factors affecting the price of agricultural products are multidimensional and uncertain, so a comprehensive analysis of the factors affecting the price of agricultural products is very important. At the same time, the factors affecting the price of agricultural products are not static; they are a dynamic process. For example, last year's garlic price was affected by a large number of hoarding by traders, and the price skyrocketed. This year's price increase is due to the reduction of garlic production due to natural disasters. Moreover, for the same influencing factors, there are also differences in the impact on different agricultural products. Therefore, a comprehensive analysis and understanding of the influencing factors of agricultural product prices is the key to improving the accuracy of agricultural product price prediction. Only by ensuring that the dimensions of the influencing factors and the amount of training data are comprehensive and accurate, the final prediction can be more accurate. In the process of growers choosing planting according to the future price trend, it is a process in which supply and demand interact with each other. Using the influencing factors of the previous year to construct a prediction model corresponding to the price of the next year, it is helpful to guide the growers what to plant. The number of species is very important.

Among the factors affecting the price of agricultural products, supply and demand are an important factor that affects prices, and they are also fundamental factors. At the same time, nonsupply and demand factors such as financial and monetary factors, political factors, policy factors, and speculative factors also need to be comprehensively considered. It can be seen that the final output and price of agricultural products is formed under the combined action of these many factors, as shown in Figure 9.

Among these many influencing factors, some influence factors have a large degree of influence on prices, while others have a small degree of influence, which is also a matter of weight. How to determine the weight of this influence factor is the focus and it causes a difficulty in agricultural product price forecasting.

### 4.3. Framework of Agricultural Product Price Prediction Model Based on BP Neural Network

The fluctuation of the price of agricultural products is mainly restricted by the basic factors of the general law of supply and demand. In addition to the basic factors, there are also factors such as weather, policies, and currency that will affect the price. The magnitude of the influence of these factors varies with time and has a certain nonlinear correlation.

The BP neural network has a strong nonlinear mapping ability. By training and learning historical price data, it is possible to find out the laws in these historical data and finally determine the degree of influence of many influencing factors on the price of agricultural products, that is, the weight of the influence.

The BP neural network uses the sigmoid function as the activation function, which has a good nonlinear mapping ability and can solve the problem of agricultural product price prediction under the influence of many factors. Among them, these influencing factors are equivalent to independent variables, such as production planting volume, production cost, import and export volume, exchange rate, rainfall, and cultivated land area. The price of agricultural products is equivalent to the dependent variable. As shown in Figure 10, the price of each period is determined by various influencing factors.

BP network (backpropagation network), also known as backpropagation neural network, through the training of sample data, constantly corrects the network weights and thresholds to make the error function drop along the negative gradient direction, approximating the desired output. It is a widely used neural network model, mostly used for function approximation, model recognition classification, data compression, and time series prediction. There are two modes of BP neural networks for forecasting: one is based on regression analysis forecasting method and the other is based on time series forecasting method. Since the agricultural products in the regional economy are obviously temporal, we adopt the forecasting method based on time series. The modeling process of the time series-based forecasting model is basically similar to the modeling process based on regression analysis, but it is not necessary to determine the influencing factors. Its basic idea is to train the network and learn the development law of time series through continuous training of time series historical samples, so as to use this law to predict its future development trend.

This paper proposes a multidimensional time series forecasting method based on BP neural network that integrates time series analysis and regression analysis. The influencing factors of agricultural product prices are used as independent variables and as input variables, and the final agricultural product prices are used as dependent variables as output. The method of variable forward shift uses the independent variable (influencing factor) of the agricultural product planting point to correspond to the dependent variable (price) of the agricultural product output time and trains and learns the historical data through the BP neural network until the convergence error is satisfied, and finally the input is obtained. The connection weight *w* is between the layer to the hidden layer and the connection weight *v* is between the hidden layer and the output layer. Using the weights obtained from training, you can input new samples to make predictions. The agricultural product price prediction model based on BP neural network is shown in Figure 11.

As can be seen from Figure 12, from 2012 to 2015, of which forecasts for 2012, 2013, and 2015 are higher than the actual values, while the 2014 data are basically the same, which shows that the actual values are very close to the forecasts. The BP neural network can basically predict the future trend of agricultural products (Shandong garlic as an example), its prediction accuracy rate is over 95%, and a very good prediction effect has been achieved.

By studying the factors affecting the price of agricultural products and using BP neural network to build a price prediction model to predict the price of agricultural products in the future, for agricultural practitioners, not only can they avoid the risks brought by the fluctuation of the agricultural product market, but also they can predict future prices by predicting the price of agricultural products, deciding what and how much to plant in the future. For the government and relevant departments, it can guide the macroeconomic policies of the regional economy and take timely and effective measures, means, and policies to carry out macrocontrol on the agricultural product market, which is of great significance to the stability of the agricultural product market.

## 5. Conclusion

The application of big data technology and the optimization of functions such as cloud computing can play a role in guaranteeing the results of data analysis. Scientific data analysis methods can have accurate data; data are a valuable information resource, which plays an important role in the development and decision management of enterprises. A large amount of agricultural data comes from a wide range of sources, and the data type is no longer a single structured data in the past, but a collection of structured data, semistructured data, and unstructured data. In order to process these complex data types, it is first necessary to preprocess them, extract relationships and entities from them, associate and aggregate them, and use a unified structure to store these data. For example, the data obtained by sensors in the agricultural Internet of Things have different formats, and a unified format is required for further processing. Among these large amounts of raw data, some data are not what we care about, which requires filtering and “denoising” to extract valid data.

Under the background of big data research, this paper takes the agricultural economy in the regional economy as the research object; studies the formation mechanism of agricultural product prices, the law of price fluctuations, and the main factors affecting agricultural product prices; and studies the methods and models of agricultural product price forecasting, innovatively combined with the characteristics of the production cycle of agricultural products, to put forward a model framework of agricultural product price prediction based on BP neural network. According to the predicted results, the macrocontrol of the industrial economy can be carried out in time to promote the healthy and stable development of the regional economy.

## Figures and Tables

**Figure 1:** Big data technology application framework.

**Figure 2:** 4V characteristics of big data.

**Figure 3:** Composition of industrial economic information model.

**Figure 4:** Flow chart of agricultural big data analysis.

**Figure 5:** Data mining flow chart.

**Figure 6:** Artificial neuron model.

**Figure 7:** The closed-loop production chain from agricultural big data to agricultural product price prediction.

**Figure 8:** Schematic diagram of planting decision points and output points in garlic price trends.

**Figure 9:** Factors affecting agricultural prices.

**Figure 10:** The price trend of agricultural products under the influence of factors.

**Figure 11:** Agricultural product price prediction model based on BP neural network.

**Figure 12:** Comparison of actual and predicted values of test results.

## Data Availability

The labeled data set used to support the findings of this study is available from the corresponding author upon request.
